# The Promotion Strategy Analysis for Green Degree of Railway Engineering Based on a System Dynamic Flow Diagram

**DOI:** 10.1155/2022/2579922

**Published:** 2022-07-14

**Authors:** Juanjuan Tang, Mengjun Wang, Xiaoying Tang, Zheng He

**Affiliations:** Department of Engineering Management, School of Civil Engineering, Central South University, Changsha 410075, China

## Abstract

This article made a system dynamics flow diagram (SD flow diagram) to describe the green railway engineering (GRE) system, which provides a theoretical basis for discussing the source and change process of the green degree of railway engineering(GDR) and also provides a practical basis for accurate policy implementation and evaluation promotion of GRE management. Based on the definition of GDR and using “input-output” relationship to analyze system structure of GRE, set two green goals of environmental and resource cost decreases as the clue, deconstructed practice process based on the principle of construction to form GRE system dynamic flow diagram, which aims to reveal the key influencing factors and promotion path of GDR. The results of the research show that (1) the green schemes set the foundation of GDR, including 3 schemes of green planning, green design, green construction, and determine the expected control values (*V*_*E*_) of 4 status, namely ecological damage degree, environmental pollution degree, land occupation degree, and resources consume degree. (2) The deviation of expected control values (*V*_*E*_) and actual control values (*V*_*A*_) from 4 status is the premise of whether the GDR needs to be optimized or improved, and 2 practice achievements of green knowledge innovation and green culture creation provided different promotion paths for GDR. (3) According to the SD flow diagram constructed by research, the 3 schemes are influenced by regional ecological carrying capacity, social material resource reserve, green knowledge reserve, green talent reserve , reasonable goals setting, strengthening preliminary research, making full use of resources, deepening the connection of procedures, and so on are conducive to build a foundation for GDR. (4) The 4 status are directly controlled by seven rate variables, which promote the dynamic optimization of GDR by technology, equipment, institution management, and behavior management. The SD flow diagram of GRE provides 2 contributions. The first provides an analytical basis for the study of the promotion strategy of GDR, and the second provides a model basis for further quantitative study of GDR.

## 1. Introduction

In the modern transportation system, the railway had green advantages in large capacity and low carbon and is still in the development stage [1, 2]. Railway construction activities bring negative environmental impacts [3], like resource and energy consumption, pollution and waste discharge, ecological landscape cutting, and destruction [4, 5], etc. At the same time, the railway product can bring positive environmental impacts, including direct benefits such as green corridor construction, the outstanding effect of land saving, energy-saving and emission reduction, and indirect ecological benefits such as innovation and upgrading of environmental protection technology and optimization of land development pattern [6]. The fundamental purpose of green railway engineering (GRE) [7] is to alleviate or absorb negative ecological effects and improve or expand positive environmental effects. Based on the long-term engineering practice, amounts of measures have been summarized or innovated, which can solve the negative environmental impact of railway construction, including clean energy use, renewable resources use, waste reduction [8], the active degradation of waste discharge standards, avoiding ecologically sensitive areas, planning vegetation system, setting up biological channels, and so on [9]. However, it is easy to ignore the economy [10] and standardization [11] of green governance under the guidance of the current evaluation index that focuses on results rather than process. At the same time, the current green evaluation index system has vague cognition and in-systematic of the green innovation and does not highlight the positive environmental effect and contribution subject of green innovation. Otherwise, the incentive effect of evaluation is not good.

Therefore, it is necessary to construct a new GDR index to reflect the green governance effect from whole process, deconstruction GRE system to reveal the practice process, and clear key factors and their responsibility body of GDR in order to provide theoretical basis to solve such problems as the economy, standardization, systematization, and incentive.

## 2. Literature Review and Concept Definition: Green Degree of Railway Engineering (GDR)

Green degree was early applied in the field of mechanical engineering and was defined as “a comprehensive evaluation index for the input of resources and energy, the output of environment and the friendliness of these inputs and outputs to the environment in the whole life cycle of a product” [12]. As the concept spread of sustainable development, the concept of green degree is widely used in other fields, such as a green degree of chemical process, the green degree of enterprise, the green degree of the supply chain, and so on. There are also some green degree studies in the field of engineering construction, and related concepts are shown in Table 1.

There are two common points in the above concepts: first, “green degree” is a concept to measure the comprehensive achievement of green goals of something; Secondly, quality, environment, and resources are the core elements of “green degree.”

There are also two weaknesses: First, although most definitions emphasize the premise of “whole process” or “whole life cycle,” each concept essentially reflects a static final result and lack of attention to the process of achieving the process and the changing rules. Second, from the perspective of green degree index content, it mainly reflects the specific needs of green goals while lacking the disclosure of essential elements.

System dynamics is widely used to solve complex and dynamic problems in construction management [18], such as construction waste reduction mechanism research [19], construction risk management research [20], and so on. The GDR is a composite concept composed of different indicators, which have different cause mechanisms and variation trends and have cross-influence in practice [21]. Therefore, the SD method also can be applied to explore the change process of GDR.

Based on the environment-economy large-scale system model [22], the natural environment is the support system for the normal operation of the social economy, mainly inputting resources into the economic system and absorbing the wastes produced by the economic system. Based on the recycle economy theory [23], renewable resources can effectively supplement the resource demand of the economic system, thus reducing the demand for natural resource exploitation. Therefore, environmental protection and resource conservation are the essential needs of the green goal. Based on the concept consensus and research weaknesses of “green degree,” “green degree of Railway Engineering” (GDR) is defined as “the comprehensive reaching effect of environmental protection and resource conservation in the whole process of railway engineering construction,” which aims to reflect the practical process of a railway engineering project and the fitting degree with expected of engineering product.

This concept emphasizes the requirement of measuring GDR both from the actual control value (*V*_*A*_) and the expected control value (*V*_*E*_) of the green target, while further analysis of the green object remains to be solved. Generally speaking, environmental protection is embodied in controlling and reducing environmental costs, including natural ecological protection (such as green corridors [24]) and pollution control of engineering activities. Resource-saving is reflected in the control and reduction of resource cost, including the optimization of land occupation (such as the combination of permanent and temporary [25], the integration of station and city [26]) and the control of production consumption (resource utilization of tunnel dregs [27]). Refer to *the Code for Environmental Protection Design of Railway Engineering* (TB 10501-2016), *Evaluation Standard for Green Railway Stations* (TB/T 10429-2014), *evaluation Standard for Green Construction of Construction Engineering* (2018 Draft for Comments), etc., the classification of GDR indexes is shown in Figure 1.

As shown in Figure 1, the ecology protection index is aimed at the natural elements, such as animals and plants, water and soil environment, geological environment, etc. Habitat cutting and secondary disasters are the prominent characteristics of linear engineering environmental impact. Pollution regulation focuses on engineering construction pollutants, such as noise, dust, solid waste, wastewater, and others, which have similar characteristics to other civil engineering construction pollutants, but the generated engineering waste components have their own characteristics [28]. The land resources index is targeted at the carrier of engineering and construction activities, the control of land resources occupation is a prominent feature of linear engineering, while the occupation optimization of large temporary engineering is a prominent feature of railway engineering [29]. The production resource index is aimed at the control of consumable resources needed for construction and production; railway engineering has outstanding characteristics in resource consumption and mechanical energy consumption [29].

## 3. The Destructive for GRE System: Based on the “Input-Output” Relationship

GRE system is an “input-output” system. The input elements included green knowledge system, green talent system, material resource system, and natural ecosystem, which is constructed and produced by engineers and takes the new artificial natural system as the main output target. The relationship is shown in Figure 2.

### 3.1. Input Elements

Inputs can be divided into 4 systems: (1) Green knowledge system is a knowledge collection required by GRE practice, such as geological and hydrological exploration data besides the line regional, environmental impact assessment report, green environmental protection technology, and so on. It is the basis for green schemes [30] formulated by participants, which mainly include green design scheme, green construction scheme, and green planning scheme, as shown in Table 2. (2) Green talent system is a collection of all kinds of talents required by green engineering practice, which has a certain identity with the green knowledge system. (3) Natural ecosystem is the carrier space of engineering practice, including geology, hydrology, flora, and fauna, etc. (4) Engineering resource system is a collection of resources required by engineering practice, including capital, raw materials, energy, and so on.

### 3.2. Output Elements

The actual output can be divided into 1 system and 3 products, which are related to the socioeconomic system, green knowledge (talent) system, and material resource system, respectively. (1) The combination of railway engineering entities and the natural environment forms a new artificial natural system, which plays a service role in the socioeconomic system and is the core purpose of engineering practice; (2) based on engineering innovation, new green knowledge (such as principle, process, technology, system, etc.), new green culture, can be produced to enrich the content of green knowledge system and train new green talents at the same time; (3) all kinds of wastes (such as wastewater, waste gas, waste materials, dust, hole slag, etc.) are generated by the construction of the project, part of the recyclable substances supplement (or exchange) the reserves of the engineering resource system through recycling and utilization, and the rest are directly emission into the natural ecosystem after degradation treatment (or removed from the region).

### 3.3. Engineering Practice System

Engineering practice system whom Linked inputs and outputs are a subjective active system based on the design and construction unit's own resources (talent team, engineering equipment, technical reserve, etc.) and is also a key part to determine the GDR, so it is the object of further research. From the spatial characteristics, railway engineering is a linear layout, and its construction organization usually divides the project into sections and pushes forward in one direction within a certain project. From the engineering management characteristics, railway construction projects are uniformly managed by construction units, and reliable and applicable advanced technology construction methods will be promoted across the whole line, thus promoting technological upgrading by comprehensive. Therefore, in the engineering system, a feedback path based onstage status assessment can be established, and an iterative upgrade of green elements in engineering system can be realized based on this path, as shown in Figure 3.

## 4. Model Construction: Based on the System Dynamic Method

### 4.1. System Boundary and Object Analysis

Based on the structural relationship of the GRE system (Figure 2), the engineering practice system is the main object to be deeply studied. It takes project approval as the starting point, completion acceptance as the endpoint, and railway engineering enterprises as the main body, involving three stages of planning, design, and construction. Each stage has different leaders and core stakeholders [33], which are different from stakeholders of other professions [34]. From the nature of work at each stage, green planning and green design only provide corresponding schemes but have not entered into engineering practice yet. Green construction involves two different works of different natures, namely scheme formulation and concrete implementation. All formulated schemes provide guidance for the concrete implementation of engineering projects, as shown in Figure 4.

Based on Figure 1, the corresponding problems are ecological damage, environmental pollution, land occupation and resources consumption, etc., which are the main observation objects of GRE. Based on Figure 3, the control values of the above green observed objects are given by the green schemes, as shown in Figure 5.

As shown in Figure 5, there are some detailed explanations.

Ecological damage reflects the destruction of the original ecosystem elements during construction, such as roadbed excavation, vegetation removal, and opening up of active areas, which usually leads to soil erosion, animal and plant diversity damage, and secondary disasters are more likely to be caused by extreme climate or geological activities [35]. Most of these activities occur in the construction preparation stage (such as temporary engineering) and also exist in the construction and production stage, such as tunnel excavation, bridge pile foundation, and excavation of abandoned soil fields. The observation of “ecological damage degree” is to ensure that the engineering activities are within the controlled range of natural carrying capacity, will not cause irreversible ecological harm (such as desertification, loss of biodiversity, etc.), and reduce the difficulty of ecological restoration.

Environmental pollution reflects the production and emission of pollutants, major pollutants including wastewater [36], waste gas emissions (from mechanical), dust, solid waste, living garbage, and so on, mainly caused by water pollution, soil pollution, air pollution, and other issues. This kind of activity runs through the whole construction process, but there are differences in environmental hazard degree and recyclable characteristics of various pollutants [37], which need to be classified and discussed. “Environmental pollution degree” is measured to ensure that emissions are within the limits of the natural carrying capacity [38] and do not incur high remediation costs (such as fines).

Land occupation is one of the focal points of the contradiction between development and protection, and the railway engineering has an important impact on the areas related to ecological security [39], such as nature reserves, cultivated land, and so on, such as cutting and occupation from the ecological perspective, and regional industrial planning from the economic perspective. Land issues focus on permanent occupation and temporary occupation. The former focuses on intensive land use (station) and land saving (line), and the latter focuses on the restoration of land function and permanent-temporary integration (construction and development cooperation). The observation of “land occupation degree” is to control the occupation amount of construction land within the approved scope of project construction land so as not to cause more than expected occupation situation, and at the same time, to timely summarize the key measures conducive to land saving (such as replacing roads with Bridges) and promote as appropriate.

Resource consumption is one of the concerns of the global resource and energy crisis and also the key point of cost control. Resources include raw materials (sand, cement, steel, etc.), energy (oil, electricity, etc.), water, etc. Construction production needs to consume a huge amount of raw materials, while many reasons will cause resource loss like engineering technology, mechanical efficiency, materials transportation, process management, and so on. The resource loss not only produces a large amount of waste but also affects ecological security. The observation of “resource consumption degree” is to ensure that the consumption degree of production materials is within the scope of the resource use plan. On the one hand, the overconsumption behavior [40] is found in time, and the response is made to avoid the delay phenomenon caused by the shortage of production materials [41]. On the other hand, summarize the key measures conducive to resource-saving (such as intelligent control, process optimization, etc.) and promote them as appropriate.

### 4.2. Causality Analysis

There are two types of causality in the causality diagram. One is the “strong to strong” positive influence relationship, which is represented by the symbol “+,” The variable *B* pointed to by the arrow will have the same change direction as the variable *A* sent by the arrow (*A* increases, *B* increases too). The other is the “strong to weak” or “weak to strong” negative influence relationship, denoted by the symbol “−,” the variable *B* that the arrow points to will have the opposite change direction with variable *A* sent by the arrow (*A* increase, *B* decrease). The causality arrow line mainly represents the direction of knowledge flow, information flow, and material flow.

#### 4.2.1. Overall Causality of GRE System

Combined with Figures 3 and 4, draw the causal diagram of the GRE system. (1) Green demand is the starting point of practice. On the one hand, it comes from ecological environment conditions and is negatively related to ecological environment carrying capacity. On the other hand, it comes from green development policy and is positively correlated with policy requirements. (2) Green scheme is the concrete implementation of green demand, mainly based on the current resource conditions, knowledge reserve, and talent reserve to make a scheme, including green design scheme and green construction scheme;. At the same time, the green scheme is a knowledge product, and the knowledge blind spot will lead to the demand for green innovation so as to realize the optimization and adjustment of the green scheme. Knowledge blind spot is negatively correlated with the total amount of green knowledge reserve. (3) Construction production is the practical application of the green scheme, so the green degree of construction production is positively correlated with the green scheme. However, due to subjective and objective reasons, the actual situation is different from the expected plan. When the green degree of construction production cannot meet the expected plan, the demand for knowledge innovation and cultural creation will be stimulated. Among them, knowledge innovation is conducive to the optimization and adjustment of green schemes, while cultural creation is conducive to the cultivation of green culture with leadership, affinity, and cohesion, so as to stimulate green construction behavior. (4) Finally, the practical result is the common result of green scheme and green construction production, which is conducive to improving ecological environment carrying capacity, increasing green knowledge reserve, and cultivating new talents with green consciousness and knowledge. The causal relationship between the above elements, the feedback loops involved, and their polarity is shown in Figure 6.

Because the negative feedback loop has a clear observation point and adjustment means, the balance can be achieved through feedback adjustment, while the positive feedback loop cannot achieve balance but can only promote its benign development through subjective initiative, and this benign development is the key to further promote the green degree of engineering. In Figure 6, green knowledge reserve and green talent reserve are the keys to the positive feedback loop, and the green degree of construction is the key to the negative feedback loop.

#### 4.2.2. Causality of Green Construct Production Process

Further analyze the production practice of green construction to understand the observation object of green construction and its causal relationship. Based on Figure 5, ecological damage degree, environmental pollution degree, land occupation degree, and resource consumption degree are analyzed.

Ecological damage is the result of demolition. The purpose of demolition is to prepare engineering carriers and work sites for engineering construction activities, mainly including site preparation, pile foundation excavation, tunnel excavation, soil collection, and abandonment, etc. Engineering wastes (such as tunnel dregs and surface soil, etc.) will be produced in the demolition process. Therefore, the ecological damage degree depends on the implementation of the established design scheme and construction scheme. For pile foundation excavation, the excavation area is determined by the design scheme, and the disturbance of excavation to the surrounding environment is determined by the construction scheme, and the control value of damage degree is determined by the established design scheme and construction scheme. When the ecological damage degree reaches or exceeds the damage control value, measures should be taken according to the situation to optimize and adjust the construction scheme or demolition behavior so as to ensure the control of the degree of ecological damage. The causal relationship is shown in Figure 7.

Environmental pollution during the construction period is the result of the discharge of nondegradable pollutants in the construction and production, so the environmental pollution degree depends on the deviation between the pollutants produced and the abatement result in the implementation of the established construction scheme and has nothing to do with the design scheme. Due to the limited capacity of the natural ecosystem to absorb pollutants, it is necessary to control the total amount of pollutants to protect the normal function of the ecosystem. The control value is based on the setting of ecological environment carrying capacity and will be reflected in the construction plan. When the environmental pollution reaches or exceeds the pollution control value, measures should be taken according to the situation to optimize and adjust the construction plan or production behavior, curb pollution discharge or strengthen pollution control so as to ensure the control of environmental pollution. The causal relationship is shown in Figure 8.

Land is the carrier of engineering and the site of construction activities. The permanent occupation of land resources is the result of the construction of engineering entities, while the temporary occupation is the result of the temporary construction of engineering production. The total occupied area is determined by the design scheme. After the completion of the project, the temporary land needs to be restored to its original function or converted to other uses, which is mainly reflected in the construction plan. The scope of construction land approved by the state sets the control value for the occupation of land and resources, which is also reflected in the design scheme. With the advancement of construction and production, green awareness and green knowledge are more abundant, or the actual occupation degree is out of control, it is necessary to carry out dynamic adjustments of the design and construction scheme according to the situation. The causal relationship is shown in Figure 9.

Resource consumption is the inevitable result of construction production. In the process of transforming materials into engineering entities, engineering waste will inevitably be generated. The consumption of engineering resources is determined by the design scheme, while the rate of material loss is affected by the construction scheme. In addition, part of the engineering waste (hole residue, waste water, etc.) generated during engineering practice can be recycled and used to supplement production materials. When the consumption of production materials reaches or exceeds the consumption control value, measures should be taken according to the situation to optimize and adjust the construction plan or production behavior so as to control the consumption of resources. The causal relationship is shown in Figure 10.

The above causality includes both a positive feedback loop and a negative feedback loop, in which all the factors leading to the deterioration of the observed object (deteriorating factors) exist in the positive feedback loop, and the balance cannot be achieved. The factors that improve the observed object (the improvement factor) all exist in the negative feedback loop, and the balance can be achieved. This suggests that aggravating factors are more important to be controlled than improving factors.

### 4.3. Parameter and Equation Design

Based on causality analysis and system dynamics (SD) parameter types, the design parameters of the GRE system are shown in Table 3.

Based on the character of different SD parameter types, the correlation between parameters is shown in Figure 11. That is, the level variable is the core observation object of the system. Rate variables directly control level variables. Auxiliary variables can affect rate variables or be constructed based on needs. The influence of external variables on the system is mainly exerted on auxiliary variables and is not affected by internal variables.

Therefore, according to the character of variables and their causality, the following parameter equation can be constructed:

1. Level variable equation
2. Notice: *T* is the construction duration of a complete project or a relatively independent partial project (such as a bridge), which is determined according to the observation range of the research object.
3. Rate variable equation
4. Notice: *f*(*x*) only reflecting the functional relations of different variables, the equation expressions need to be determined on the basis of further research, which is not in the scope of this paper.
5. Auxiliary variable equation
6. Notice: *g*(*x*), *u*(*x*), *h*(*x*) only reflects the functional relations of different independent variables, and the equation expressions need to be determined on the basis of further research, which is not in the scope of this paper. Since there is some information delay between green knowledge innovation and scheme optimization adjustment, the function “SMOOTH” is used to simulate the effect of information delay, and “stime” is used to show the delay time.

(1) $$\begin{array}{c} \left\{\begin{array}{c} L_{i}=\int_{t=0}^{T}R_{i1}\text{d}t-\int_{t=0}^{T}R_{i2}\text{d}t,\;i=1,2,3,\\ L_{4}=\int_{t=0}^{T}R_{4}\text{d}t. \end{array}\right. \end{array}$$

(2) $$\begin{array}{c} \left\{\begin{array}{c} R_{i1}=f_{i}\left(A_{1},A_{22}\right),\;i=1,2,4,\\ R_{31}=f_{3}\left(A_{1}\right),\\ R_{j2}=f_{j}\left(A_{1}\right),\;j=1,2,3. \end{array}\right. \end{array}$$

(3) $$\begin{array}{c} \left\{\begin{array}{c} A_{1}=g_{1}\left(E_{1},E_{2},E_{3},E_{4},\text{SMOOTH}\left(A_{21},\text{stime}\right)\right),\\ A_{1i}=g_{i+1}\left(A_{1}\right),\;i=1,2,3,4, \end{array}\right. \end{array}$$

### 4.4. SD Model for GRE Practice Process

On the basis of parameter definition and causality, the system dynamic flow diagram is established to reflect the overall practice process of GRE and also reflect the changing process of GDR, as shown in Figure 12.

## 5. Results and Discussion

### 5.1. The Characteristic Analyses for GRE Practice Process

As shown in Figure 12, the important characteristics of GRE practice can be analyzed through the nature, position, and interaction between variables. With state variables as the center, this paper expounds on the causal relationship, feedback link, critical path control, and other aspects successively.

#### 5.1.1. Give Priority to Controlling Deteriorate Factors: *R*_11_, *R*_21_, *R*_31_, *R*_41_

On the one hand, the deteriorate factor is preaction, and the improvement factor is postaction. Preaction control has significant advantages over post-action disposal, which is also conducive to cost control. On the other hand, the loop where the deteriorate factors are located is a mainly positive feedback loop, which will lead to the deterioration or even collapse of the system, like the out of control in cost or irreversible ecological damage at the worst.

#### 5.1.2. Control Value Setting and Level Variable Observation Determine the Effectiveness of Feedback Mechanism: *A*_11_∼*A*_14_, *L*_1_∼*L*_4_

The control value (*A*_11_∼*A*_14_) is reflected in the green scheme (*A*_1_), which needs to maintain a certain stability. However, with the deepening of practice and the increase of cognition, there is also an objective, practical need for optimization and adjustment, but there is an upper limit to protecting environmental carrying capacity so as to maintain the self-regulation function of the ecosystem. Level variables (*L*_1_∼*L*_4_) usually reflect the actual situation, but due to the need for prevention and management, prediction and judgment should be made based on their development rules so that measures can be taken in advance to control or reverse the deterioration trend in time.

#### 5.1.3. Significant Gathering Points that Control the Critical Path: *A*_1_, *A*_21_, *A*_22_

The name of 3 points can be found in Table 3. They are green scheme (*A*_1_), the function gathering point of exogenous variables and internal variables of the system; green knowledge innovation (*A*_21_) and green culture creation (*A*_22_), the aggregation point that makes up the feedback loop. According to its location and direction of the arrow line, the green scheme is the green foundation of GDR, while green knowledge innovation and green culture creation are the key factors to improving GDR.

#### 5.1.4. Two Kinds of Improving Path: by A_21_ and A_22_

Firstly, green knowledge innovation (*A*_21_) can promote the optimization and adjustment of the green scheme to improve the GDR, which is the all-around “quality” improvement (*L*_1_∼*L*_4_). However, there is a delay effect in this path, mainly because there is a process of demonstration and promotion in the practical application of green knowledge innovation results. The second is to improve the GDR by promoting the optimization and adjustment of some deteriorate factors (*R*_11_, *R*_21_, *R*_41_) through green culture creation (*A*_22_), which is the improvement of targeted (*L*_1_, *L*_2_, *L*_3_) “quantity” without delay effect.

#### 5.1.5. Planning and Initiative Are Necessary for GDR Improving: *E*_3_, *E*_4_, and *A*_31_∼*A*_34_

Green knowledge innovation and green culture creation are influenced by two kinds of system parameters. In terms of green knowledge innovation (*A*_21_), real-time innovation caused by deviation (*A*_31_∼*A*_34_) has a longer delay effect. The planned innovation based on the weakness of green knowledge reserve (*E*_3_) can make full use of the noncritical path of schedule arrangement and shorten the delay effect of achievement application effectively. As far as green culture creation (*A*_22_) is concerned, the demand for green culture based on the diverse consciousness of green talent reserve and the unified ideology is more comprehensive and can be gradually deepened and assimilated with the engineering practice. The demand for immediacy culture caused by the deviation is more targeted and can effectively supplement the green culture of the project.

In general, the GRE practice process based on system dynamics modeling further reveals the core of the green target is to control ecological damage, environmental pollution, and optimization of land occupation and promote the resource-saving. The key link of control is condition monitoring; a green scheme sets a good foundation for the GDR, and green knowledge and green culture promote GDR improvement through two kinds of paths, respectively.

### 5.2. The Promotion Strategy for GDR

Based on the analysis of characteristic in Section 5.1.4, the GDR promotion strategy is mainly proposed from two aspects of source optimization and dynamic optimization. The former strategy comes from characteristic in Section 5.1.5, while the latter strategy comes from characteristic in Section 5.1.1.

#### 5.2.1. Source Optimization Strategy for GDR

Source optimization takes green scheme optimization as its main target and is realized by controlling or optimizing its influencing factors. The causes tree of *A*_1_ is shown in Figure 13.

Green schemes include green design scheme, green construction scheme, and green planning scheme (Table 2), which lay a foundation for the GDR from three aspects of green function, green implementation, and green support, respectively. Relevant source optimization strategies are shown in Table 4.

#### 5.2.2. Dynamic Optimization Strategy for GDR

Dynamic optimization is realized by controlling or optimizing the influencing factors of the green observation object. The causes tree of Level variables and deviations is shown in Figure 14.

Since the Level variable is only controlled by the rate variable, the dynamic optimization strategy of the Level variable is mainly proposed from the deteriorate factor and improvement factor. The Rate variable depends on two factors: construction scheme guidance and construction behavior management. The specific dynamic optimization strategy and its target are shown in Table 5.

Starting from the purpose of “Promote construction through evaluation,” the above 3 schemes and 4 Level variables should be set as an evaluation index, and the corresponding promotion strategy can be refined into secondary indicators, which can enrich the existing index system to a “source—process—result” indicators cover the whole process and make a comprehensive evaluation of GRE.

## 6. Conclusions

Lack of attention to dynamic process in the engineering practice is a problem in existing green evaluation index system, which caused a research interests in change mechanisms of GDR and constructed the GRE dynamics model to make clear the 3 sources and 2 promotion paths of GDR, in order to put forward targeted strategy to GDR promotion from classification management idea. The main contents and significance include the following:

1. Through the definition of the concept of GDR, we clearly defined the measuring method of relative value (control value, actual value) in the whole process for the green degree. Although the GDR index has the possibility of imperfection, the main significance is to break the limitation of a static description of green degree by the absolute final value in the past;
2. Simplify and deconstruct the GRE system structure based on the causality of “input-output,” clarify the primary and secondary objectives of engineering practice through the cognition of the relationship between various parts, and further focus on engineering practice system to determine the research boundary range of GDR, to put forward the necessity of dynamic improvement research for GDR;
3. Based on the boundary and object analysis of GRE, establish the overall system causality diagram firstly according to the principle of construction procedure, then focus on 4 aspects including ecological damage, environmental pollution, land occupation, and resources consumption to establish causality diagram severally. According to the characteristics and the causal relationship between the factors, the parameter classification and equation were designed. Thus, the dynamic flow diagram of the GRE system is formed to clarify the source and optimization path of GDR.

There are still some deficiencies in this study, and the key problem is that there is no further verification of the system dynamics model. However, the purpose of this paper is to analyze the dynamic relationship between the GDR index of railway engineering and its influencing factors, which is a reasonable abstraction based on reality, and model verification is the prerequisite of simulation. Therefore, the core of this study is to construct the system dynamics flow diagram and propose the strategy for improving the GDR through the interpretation of the flow diagram, which not only puts forward the data support requirements of GDR management but also puts forward the improvement direction for the precise governance and intelligent improvement of green goals. In the future, based on the system dynamics flow diagram constructed in this paper, further quantitative research on the GDR will be carried out. Through model verification, optimization, and simulation, the change trend of the 4 status of green observation objects will be grasped so as to formulate targeted intervention control strategies, implement expected management, and improve engineering management benefits.

## Figures and Tables

**Figure 1:** Classification of GDR indexes.

**Figure 2:** Structure and relationship of GRE system.

**Figure 3:** Dynamic optimization process of GRE practice based on PDCA process.

**Figure 4:** Realization process of GRE.

**Figure 5:** Green observation objects and observation purpose of GRE practice system.

**Figure 6:** The causality of the GRE system.

**Figure 7:** The causality of ecological damage degree.

**Figure 8:** The causality of environment pollution degree.

**Figure 9:** The causality of land occupation degree.

**Figure 10:** The causality of resource consumption degree.

**Figure 11:** The correlation between SD parameters.

**Figure 12:** A SD flow diagram for GRE practice process.

**Figure 13:** The causes tree of the green scheme (*A*_1_).

**Figure 14:** The causes tree of level variables (*L*_1_∼*L*_4_) and deviations (*A*_31_∼*A*_34_).

**Table 1:** Definition and evaluation indexes of various green degrees in the engineering construction field.

Name	Definition	Evaluation index
Green degree of building	Evaluation criteria used to describe the degree of harmony between buildings and the environment and the degree of construction rationalization [13]	Safe and durable, healthy and comfortable, convenient life, resource-saving, livable environment [13]

Green degree of highway	In the whole life cycle, adhere to the concept of green development, protect the ecological environment, improve the quality of the project, save intensive resources and improve the degree of service quality [14]	Green concept, ecological environmental protection, resource conservation, quality construction, service improvement [14]

Green degree of construction	In the whole process of construction to achieve green development, low-carbon environmental protection, resource cycle of the green degree [15]	Energy resources, environmental protection, construction management, technological innovation, and social coordination [15]

Green degree of materials	It is used to measure the applicability of sand concrete with different litho logic mechanisms to railway engineering in complex and dangerous mountainous areas [16]	Performance, economic benefits, social benefits, environmental impact, production technology [16]

Green degree of temporary facilities	The degree of energy-saving, environmental protection, turnover, and efficient production in the whole life cycle [17]	Balanced ecological environment, scientific space layout, reasonable construction economy, coordinated management, and operation [17]

**Table 2:** Task and content of green schemes.

Type	Task	Content
Green design scheme (including preliminary design, technical design, and construction design) [31]	Green design of engineering structure	Reduce the occupation of cultivated land, strengthen the design of disaster prevention and mitigation, improve the health and durability of the project, implement the function of energy conservation and emission reduction; taking the systematic design of engineering and environment as an opportunity to intervene in the comprehensive management of ecological restoration and promote the harmonious coexistence of engineering and human activities
	Green design of temporary engineering	Design temporary engineering from the perspectives of sustainable use of the site, permanent and temporary integration, convenient transportation, and emission reduction
	Green design of environmental protection facilities	Ensure the realization of green production in railway operation and solve environmental problems such as waste discharge management, vibration noise elimination, electromagnetic radiation barrier, and so on

Green construction scheme (construction organization design, clear resource allocation, production layout, technology, etc.) [32]	Disturbance control	Reduce the disturbance or damage to the natural environment caused by construction operations
	Resource-saving	Improve the efficiency of resource utilization and strengthen resource management
	Pollution prevention and control	Reduce the discharge of pollutants in construction operations, treat the output pollutants, and discharge them to standards
	Ecological remediation	Site restoration, planting grass, and trees, etc.
	Labor conservation and protection	Environmental protection education, environmental protection skills training, environmental protection theme activities, green operation environment construction, etc.

Green planning scheme	Green knowledge innovation plan	The establishment of scientific research projects aiming at the knowledge blind spots and difficult problems of green knowledge reserve usually depends on the needs of national scientific research plans or projects
	Green culture creative plan	In order to promote group cohesion, cultural unity action should be carried out aiming at the pluralism of group ideology of participants in engineering practice

**Table 3:** Parameter list of GRE system.

Type	Character	Name	Symbol
Level variable (*L*)	A variable that determines the behavior of the system over time. The value of the current moment is equal to the value of the past moment plus the change in time over time	Ecological damage degree	*L*_1_
		Environmental pollution degree	*L*_2_
		Land occupation degree	*L*_3_
		Resource consumption degree	*L*_4_

Rate variable (*R*)	A variable that directly changes a level variable, reflecting the speed at which the state variable is input or output	Environment damage rate	*R*_11_
		Ecological restoration rate	*R*_12_
		Pollution emission rate	*R*_21_
		Pollution treatment rate	*R*_22_
		Land occupancy rate	*R*_31_
		Release occupancy rate	*R*_32_
		Resource consumption rate	*R*_41_

Auxiliary variable (*A*)	Variables that affect the system but do not directly control the level variable have independent values at each time	Green schemes	*A*_1_
		Control values from green schemes	*A*_11_∼*A*_14_
		Green knowledge innovation	*A*_21_
		Green culture creative	*A*_22_
		Deviations form level variable	*A*_31_∼*A*_34_
		Engineering garbage	*A*_4_
		Garbage recycling	*A*_41_
		Wastage	*A*_42_

External variable (*E*)	It varies over time but not by any other variable in the system	Eco-environmental carrying capacity	*E*_1_
		Green resource conditions	*E*_2_
		Green knowledge reserve	*E*_3_
		Green talent reserve	*E*_4_

**Table 4:** Source optimization strategy of GDR.

Influence factor	Green scheme		
	Green design scheme	Green construction scheme	Green planning scheme
Environmental carrying capacity (*E*_1_)	Deepen hydrogeological survey, deepen environmental impact assessment, optimize damage control value and pollution control value standards, and determine the baseline control basis	Implement the comments on environmental impact assessment actively, and propose construction plans with less disturbance, less pollution, and faster repair	/

Green resource conditions (*E*_2_)	Apply new technology, new materials, etc. to design engineering structure, optimize occupation control value and consumption control value, and determine the baseline control basis	Apply new technology, new equipment, and other construction organization design, the development of small disturbance, low pollution, less waste, excellent treatment of the construction scheme	Set up green innovation research projects appropriately ahead of schedule

Green knowledge reserve (*E*_3_)

Green talent reserve (*E*_4_)	Increase the proportion of green designers with green knowledge and practical experience, deepen the effect of green design	The proportion of green construction personnel with rich green knowledge and practical experience should be increased to promote the group's green ideology and awareness	Overall planning of green knowledge training and education, the establishment of incentive mechanism

Green knowledge innovation (*A*_21_)	Promote and apply innovative achievements in time to optimize design schemes	Promote and apply innovative achievements in time to optimize the construction plan	/

**Table 5:** Dynamic optimization strategy of GDR.

Level variable	Influence factor	
	Deteriorate factor management	Improvement factor management
Ecological damage degree (*L*_1_)	Decrease *R*_11_: ①Optimization of construction technology based on green knowledge innovation achievements to reduce the disturbance range and frequency	Increase *R*_12_: Improve vegetation restoration ability and reduce soil erosion based on green knowledge innovation (using science and technology to protect the environment)
	②Through the green culture creation to improve the awareness of green environmental protection, reduce the damage intensity of operation behavior	

Environmental pollution degree (*L*_2_)	Decrease *R*_21_: ①Optimize construction technology and use green materials based on green knowledge innovation achievements to reduce the rate of pollutant generation	Increase *R*_22_: Based on the achievements of green knowledge innovation, the ability of pollutant collection and treatment should be improved, and the equipment and process of pollutant treatment should be innovated
	②Strengthen the management of pollution sources, establish the pollutant statistical ledger, find its statistical rules to determine the reasonable pollutant treatment threshold	
Land occupation degree (*L*_3_)	Control *R*_31_: Based on the green knowledge innovation achievements, the proportion of bridge and tunnel and the building limit of the project were optimized, and the layout scheme of temporary engineering was optimized to reduce the occupation of rare land resources	Increase *R*_32_: Based on the green knowledge innovation achievements, the proportion of permanent and temporary combination design of temporary engineering was improved, and the use conversion paradigm of temporary engineering was explored to improve the level of land resource recovery and reuse

Resource consumption degree (*L*_4_)	Decrease *R*_41_: ①The application of advanced equipment and information technology to assist production, achieve accurate discharge, and reduce the speed of resource consumption	Increase *A*_41_: Innovation of engineering waste recycling and reusing technology, improve the recovery capacity, improve the capacity of local materials use
	②Establish resource consumption and consumption ledger, optimize waste disposal and transportation plan through statistical law	

## Data Availability

No digital data were used to support the findings of the study.
